# Reduced expression of Snail decreases breast cancer cell motility by downregulating the expression and inhibiting the activity of RhoA GTPase

**DOI:** 10.3892/ol.2013.1385

**Published:** 2013-06-07

**Authors:** ALI ZHANG, QUANSHENG WANG, ZHIQIANG HAN, WEI HU, LING XI, QINLEI GAO, SHIXUAN WANG, JIANFENG ZHOU, GANG XU, LI MENG, GANG CHEN, DING MA

**Affiliations:** 1 Cancer Biology Research Center, Tongji Hospital, Tongji Medical College, Huazhong University of Science and Technology, Wuhan, Hubei 430030;; 2 Radiotherapy and Chemotherapy Department, Zhongnan Hospital, Wuhan University, Wuhan, Hubei 430000;; 3 Department of Chinese Medicine, Union Hospital, Tongji Medical College, Huazhong University of Science and Technology, Wuhan, Hubei 430030, P.R. China;; 4 Department of Gynecologic Medical Oncology, The University of Texas M.D. Anderson Cancer Center, Houston, TX 77030, USA

**Keywords:** Snail, RhoA GTPase, metastasis, breast cancer

## Abstract

Several lines of evidence support an important role for Snail, a transcriptional factor, in breast cancer. Overexpression of Snail has been associated with breast cancer metastasis, although the specific role of Snail in the process remains unclear. To address this issue, the expression levels of Snail, RhoA and fibronectin, as well as MMP-2, were reduced in the breast tumor cell lines MDA-MB-231 and MDA-MB-435S, and their biological responses were studied *in vitro* and *in vivo*. For the first time, it was observed that downregulated Snail expression is correlated with a significant inhibition of the expression and activity of RhoA GTPase, as well as MMP-2. The present data provide evidence that Snail promotes tumor cell motility and angiogenesis which is mainly mediated through the regulation of RhoA activity. In conclusion, the present findings demonstrate a key regulatory role for Snail in breast tumor growth and progression.

## Introduction

Breast cancer is the leading cause of cancer-related mortality in females worldwide (1). Primary breast cancer tumors may be removed or irradiated relatively simply, but distant metastases are difficult to treat. Tumor cell motility is the hallmark of invasion and an essential step in metastasis. One important insight came from the discovery that the increased motility and invasiveness of cancer cells is reminiscent of the epithelial-mesenchymal transition (EMT) that occurs during embryonic development (2). In this process, epithelial cells acquire fibroblast-like properties such as the functional loss of E-cadherin. Studies have shown that several transcription factors, including the Snail/Slug family (3), δEF1/ZEB1 (4) and SIP1 (5) have been implicated in E-cadherin repression. Snail, a zinc finger protein, is considered to be a critical EMT regulator (6). Although a direct link between Snail expression and tumor metastasis has not yet been reported, a number of studies have shown that the overexpression of Snail is correlated with tumor invasion (7).

Studies have shown a correlation between Snail expression and the degree of infiltration in breast carcinomas (8). Snail is also an upstream protein of metalloproteinase-2 (9), which is a mesenchymal marker sufficient to trigger EMT *in vivo* (10). Although a report has shown that RhoB, a small GTPase involved in cytoskeletal actin rearrangement, lies downstream of Slug (11), another member of the Snail super-family, there is no evidence to support a link between Snail and Rho GTPases.

Rho GTPases belong to the Ras superfamily of small GTPases and are highly conserved throughout eukaryotes. These proteins control the dynamics of the actin cytoskeleton and thus represent key regulatory molecules that are active during cell migration (12). RhoA has been implicated in the formation of stress fibers and cell adhesion in fibroblasts. A number of reports have shown that RhoA expression is upregulated in a group of malignancies (13) and that the activity of RhoA is correlated with lymph node metastasis in colorectal cancer (14). The expression level of RhoA is positively correlated with the progress of these carcinomas.

In the present study, Snail and RhoA were observed to be overexpressed in breast cancer tissues compared with normal breast tissues and the expression of Snail and RhoA was associated with the differentiation grade and lymph node metastasis of breast cancer, respectively. We hypothesized that Snail, as a transcription factor, may promote breast cancer metastasis through the regulation of RhoA expression and activity.

## Materials and methods

### Cell lines and antibodies

The breast cancer cell lines MDA-MB-231, MDA-MB-435S and human mammary epithelial cells (HMEC; Invitrogen Life Technologies Corporation, Carlsbad, CA, USA) were maintained in Dulbecco’s minimum essential medium (DMEM) supplemented with 10% FCS and 1% antibiotic/antimycotic solution. Polyclonal antibodies against Snail, E-cadherin, MMP-2 and β-actin, and monoclonal antibodies against fibronectin, RhoA, Rac1, Cdc42 and PECAM-1 were obtained from Santa Cruz Biotechnology, Inc. (Santa Cruz, CA, USA).

### Immunohistochemical staining

Conventional paraffin-embedded tissue sections obtained from breast tumors and normal breast tissue were obtained from surgical specimens resected at the Tongji Hospital of the Huazhong Science and Technology University (Wuhan, China). The avidin-biotin complex immunoperoxidase method was used to study the levels of Snail and RhoA expression by immunostaining. The frequency of each protein was scored as the percentage of positive cells as follows: negative, <5%; weak, 5 to 25%; moderate, 25 to 50%; and strong, >50%.

### Vectors and transfections

cDNA encoding the open reading frame of Snail was amplified and cloned into the pIRES2-EGFP vector (Invitrogen, Carlsbad, CA, USA) in the inverted direction to produce an antisense-Snail cDNA construct (AsSn). Transient transfection for GFP alone (mock, Invitrogen), GFP-fused forms of wild-type RhoA, dominant-negative (DN) N19-RhoA and activated (Act) V14-RhoA (kindly provided by Professor Richard Pestell, Albert Einstein College of Medicine, New York, NY, USA) were also transfected into MDA-MB-231 and MDA-MB-435S cells and were then selected using 800 *μ*g/ml G418 for 12 days. Clones were picked and expanded for an additional two months. Experiments with the transiently transfected cells were performed 72 h after the transfections.

### Real-time PCR

Total RNA was extracted according to the TRIzol instructions (Invitrogen), then combined with an RNase-free DNase kit (Promega, Madison, WI, USA) and reverse transcribed with random primers. The resulting cDNA was used for PCR using SYBR-Green master PCR mix (Toyobo, Osaka, Japan) in triplicate. PCR and data collection were performed on a M×3000P™ Real-Time PCR system (Stratagene, La Jolla, CA, USA).

### Western blotting

The protein content of each lysate was determined by a Bio-Rad protein assay (Bio-Rad, Hercules, CA, USA). Each lysate (10 *μ*g) was resolved on a 10 to 12% denaturing polyacrylamide gel and transferred electrophoretically to a nitrocellulose membrane (Amersham Biosciences, Piscataway, NJ, USA). After incubation with primary antibodies at 4°C overnight, the immunoreactive proteins were localized with horseradish peroxidase-conjugated secondary antibodies (Santa Cruz Biotechnology, Inc., Santa Cruz, CA, USA). The reactants were developed using an enhanced chemiluminescence kit (Amersham Biosciences).

### Reporter assays

The RhoA promoter sequence (−2,112 to +75 bp) was cloned into the pGL3-Basic vector (Promega, Madison, WI, USA) to be used as a reporter assay. The AsSn (or pIRES2-EGFP vector) and fly-luciferase plasmids were cotransfected into MDA-MB-231 and MDA-MB-435S cells using Lipofectamine 2000 (Invitrogen). After 48 h, firefly and Renilla luciferase activities were measured using the Dual Luciferase Reporter Assay kit (Promega).

### Cell mobility assay

For the wound-healing migration assay, ∼250,000 cells were seeded in six-well plates and grown to 100% confluence. A 10-*μ*l pipette tip was used to create a scratch down the middle of each well. Representative images were photographed using phase-contrast microscopy at the indicated times.

For the cell migration assay, 1×10^4^ cells were seeded on the top of Transwell membranes treated with Matrigel matrix (BD Biosciences, Franklin Lakes, NJ, USA) following the manufacturer’s instructions. After 10 h of incubation, filters were fixed with 4% paraformaldehyde (15 min, 4°C); the number of cells on the top surface of the filters was estimated by counting three independent visual fields using a microscope. The average number of cells in four replicate wells was determined for each cell line in each of three independent experiments.

### Cell proliferation assay

Cells (5×10^3^) were plated in 96-well plates and allowed to attach and grow in regular medium for 4 h. At each time point (0, 12, 24, 36, 48, 60 and 72 h of culture), 10 *μ*l MTT (5 mg/ml) was added to each well. The reaction was stopped after 4 h of incubation by adding 150 *μ*l dimethyl sulfoxide (DMSO). The optical density (OD) value was obtained by measuring the absorbance at a wavelength of 570 nm. The proliferation assay was performed in triplicate and repeated three times.

### GTPase activity assays

The activities of Rac1, Cdc42 and RhoA were studied as described previously (15). Glutathione S-transferase (GST)-C21 was used to detect Act-RhoA. GST-PAK-CD, a fusion protein that selectively binds to GTP-Rac1, was used to active Rac1 and Cdc42 fusion proteins was generated as described previously. Cells were lysed at 4°C in 300 *μ*l lysis buffer and then centrifuged; 15 *μ*l supernatant was kept as a total lysate control and the remaining volume was mixed with fusion proteins in the presence of glutathione-agarose beads. The mixtures were incubated for 16 h at 4°C, beads were pelleted and washed and bound proteins were eluted in Laemmli electrophoresis buffer. The proteins were resolved by SDS-PAGE on 12% polyacrylamide gels and transferred to polyvinylidene fluoride membranes (Hybond-P, Amersham Pharmacia Biotech, Amersham, UK), which were incubated with antibodies to RhoA, Rac1 or Cdc42 (diluted 1:1000).

### In vivo tumorigenicity studies

Female athymic nude mice (BALB/c nu/nu) aged between four and five weeks were obtained from the Shanghai Institute of Medical Material (Shanghai, China). Parental and AsSn-transfected MDA-MB-231 and MDA-MB-435s cells were harvested, washed, resuspended in PBS and injected into the mammary fat pad of mice. Tumor growth was measured three times each week. For survival analysis, the mice were euthanized and sacrificed when they appeared moribund. All experiments were performed at least twice, and samples from the breast tumors, lungs, liver and lymph nodes were obtained. Tissues for histological examination were fixed and embedded in paraffin using standard methods.

### Statistical analysis

Spearman’s rank tests were used to evaluate the correlation between Snail or RhoA expression and clinical pathological parameters. SPSS 16.0 software (SPSS, Chicago, IL, USA) was used to carry out all statistical analyses. P<0.05 was considered significant to indicate a statistically significant difference.

## Results

### Increased expression levels of Snail and RhoA were observed in human breast cancer tissues

The expression and subcellular localization of Snail and RhoA were studied in a set of specimens derived from 20 normal breast tissues and 60 breast cancer tissues. In the normal breast tissues examined, only faint nuclear staining for Snail and cytoplasmic staining for RhoA were detected, whereas the breast carcinomas exhibited strong staining for Snail and RhoA (Fig. 1A). To further investigate the possible correlation of Snail and RhoA expression with the progression of breast cancer, we evaluated the protein expression of Snail and RhoA in normal breast and breast tumor, and the clinicopathological characteristics in these specimens. It was found that Snail and RhoA expression significantly higher in breast cancer (Table I), and RhoA expression was correlated with differentiation grades of breast tumor (Table II). Western blotting analysis for Snail and RhoA in breast cancer and adjacent normal tissues obtained from 15 patients showed increased levels of Snail and RhoA in the cancerous tissues (Fig. 1B). These results suggest that Snail and RhoA may be involved in the progression of breast cancer.

### Gene expression involved in EM T was altered in AsSn-transfected MDA-MB-231 and MDA-MB-435S cells

AsSn was stably introduced into the human breast cancer cell lines MDA-MB-231 and MDA-MB-435S, which express relatively high levels of Snail mRNA and exhibit the invasive phenotype. A low level of Snail expression in AsSn MDA-MB-231 clones was demonstrated by western blotting with anti-Snail antibody, while Snail expression was not affected in the mock-transfected cells. A similar result was observed in the MDA-MB-435S cell line (Fig. 2A), demonstrating that the loss of Snail expression is achieved in independent clones.

Whether the introduction of AsSn affected the expression of EMT genes using western blotting analysis MDA-MB-231 was investigated. Analysis of several independent clones revealed increased expression levels of E-cadherin and a significant decrease in endogenous fibronectin and MMP-2 expression in AsSn cells, whereas RhoA expression was reduced by ∼60% in AsSn cells (Fig. 2A).

To exclude the possibility that the knockdown by the anti-sense vector was not Snail-specific, the mRNA expression level of Slug, a close homolog of Snail, was detected by real-time PCR. No significant changes in the level of endogenous Slug mRNA were detected in the AsSn- or mock-transfected clones (Fig. 2B).

Furthermore, the mock-transfected clones exhibited spindle-shaped cells and fibroblastic morphology, whereas AsSn clones typically displayed a cobblestone-like, epithelial morphology (Fig. 2C).

### AsSn alters the motility of MDA-MB-231 and MDA-MB-435S transfected cells in vitro

It was observed that the downregulation of Snail in breast tumor cells significantly reduced cell migration from the edge of the wound 24 h after scratching (Fig. 3A). Similarly, when the cell invasion potential was measured in a Matrigel-coated Transwell assay, mock-transfected and AsSn cells were observed to invade the bottom of the membrane. However, in the 10-h period, the number of migrating mock-transfected cells was three- to four-fold greater than that of the AsSn cells (Fig. 3B) and this difference persisted over a period of 24 h.

To exclude the possibility that differences in the growth rates of the mock-transfected and AsSn cells affected the interpretation of these results, cell growth was observed over 72 h and curves were plotted. There was no significant difference between the proliferation of the mock-transfected and AsSn cells after 72 h, excluding such a possibility (Fig. 3C). This result indicates that AsSn does not affect cell proliferation *in vitro*.

### AsSn downregulates the expression and alters the activity of RhoA in transfected cells, suggesting a role in invasion in vitro

A reporter construct containing the RhoA promoter was transfected into the same cells and which were analyzed for promoter activity. The transient transfection results showed a two- to three-fold repression of RhoA promoter activity by Snail downregulation, suggesting that RhoA expression was under the control of Snail (Fig. 4A).

To investigate whether AsSn was capable of inactivating Rho GTPase and whether this inactivation was involved in the decreased migration ability, GTPase assays were performed using GST fusion proteins with binding domains that bind only activated forms of these GTPases. As shown in Fig. 4B, there was a decrease in the expression level of Act-RhoA in AsSn cells compared with mock-transfected cells. By contrast, the levels of active Rac1 and Cdc42 show no difference between the AsSn- and mock-transfected cells.

To further analyze the involvement of RhoA inactivation in invasion, GFP-fused wild-type, DN (N19-RhoA) or active (V14-RhoA) RhoA vectors were transfected into the cells and the invasion ability was measured *in vitro*. A significant decrease in the invasion ability of AsSn cells was obtained with transfectants expressing DN-RhoA, whereas overexpression of Act-RhoA increased the invasion ability of the transfectants compared with transfectants expressing GFP alone (Fig. 4C). Western blotting control experiments using anti-GFP and anti-RhoA antibodies demonstrated the expression of the GTPase forms in transfected cells (Fig. 4D). Whether there was an association between RhoA and MMP-2 activation was then studied. As shown in Fig. 4E, MMP-2 expression and activity decreased in cells transfected with DN-RhoA and increased in cells with Act-RhoA.

### AsSn alters primary tumor growth and lymph node metastasis in vivo

Mice that received an injection of mock-transfected cells developed tumors of >1.5 cm in diameter (Fig. 5A) and their mean survival time was 60 days (Fig. 5B). However, mice that received an injection with AsSn-transfected cells developed tumors with a diameter of <0.5 cm (Fig. 5A) and their mean survival time was >90 days (Fig. 5B). Microscopically, no metastases were observed in the liver or lungs, although they were detected in the lymph node (Fig. 5C). Lymph node metastases developed in 80–90% of the mice injected with mock-transfected cells, whereas the mice injected with AsSn cells developed lymph node metastases in only 20% of cases. Similar results were observed with MDA-MB-435s cells (data not shown).

Western blotting analysis showed decreased levels of Snail and RhoA proteins in the tumors that received an injection of AsSn cells (Fig. 5D), compared with the control group that received an injection of mock-transfected cells.

## Discussion

In the present study, it was observed that Snail and RhoA were coexpressed at significantly higher levels in breast cancer tissues compared with normal tissues, according to immunohistochemical analyses and western blotting. Analysis of the clinicopathological characteristics (Table I) shows for the first time that Snail and RhoA protein expression is associated with differentiation grades and lymph node metastasis. We hypothesized that Snail and RhoA may be involved in the progression of malignant behavior in breast cancer and RhoA may act as a downstream target of Snail. Previous studies have suggested that Snail expression is correlated with the presence of lymph node metastases (16) and RhoA protein expression is upregulated in breast cancer tissue (17), enhancing migration and invasion in breast cancer cell lines (18). To investigate this issue, the potential role of Snail in the invasion of breast tumor cells was assessed at the molecular and cellular level, with the *in vitro* and *in vivo* metastasis properties of estrogen receptor (ER)-negative MDA-MB-231 and MDA-MB-435S cell lines transfected with AsSn and DN-RhoA or Act-RhoA vectors.

By inhibiting Snail expression, clear changes were observed in the expression of several important components of the EMT proteome in AsSn cells. The EMT proteome reflects a fundamental change in the proteins gained or lost in the transition of tumor epithelia to metastatic cells (19). Since RhoA is required for the generation of the contractile force which leads to the rounding of the cell body and is required for the regulation of microtubule polymerization in cell mobility (20), RhoA may increase cell motility. MMP-2, a candidate invasion gene, may also increase motility as it is capable of degrading the extracellular matrix and components of the basement membrane (21). In the present study, the induced protein expression of E-cadherin and decreased expression of RhoA, MMP-2 and fibronectin, a component of the extracellular matrix, were observed in AsSn-transfected breast cancer cells. Unchanged mRNA expression of Slug was also detected in AsSn cells, excluding a possible off-target effect of AsSn. These findings suggest that AsSn has an inhibiting effect on MMP-2, fibronectin and RhoA.

Cell invasion is associated not only with the ability to be motile, but also the ability to degrade the extracellular matrix. The decreased invasion ability of AsSn cells was coupled with the downregulated expression of RhoA and MMP-2, suggesting that cell motility and extracellular matrix degradation are likely to be functionally interdependent for cell invasion. We suggest that Snail may modulate RhoA expression and trigger Rho GTPase-dependent signaling, leading to the control of MMP-2 expression.

The metastasis and survival time after injection of mock-transfected and AsSn MDA-MB-231 cells into BALB/C SCID mice was further tested *in vivo*. At the end of the experiment, a significant reduction in the volume of tumors induced by AsSn cells and less lymph node metastasis was detected compared with mock-transfected cells. The results indicate that the full biological effect of blocking Snail must be markedly affected by the tumor microenvironment. Furthermore, mice injected with AsSn cells survived longer than those injected with mock-transfected cells. Significantly decreased levels of RhoA protein were observed in the tumors derived from mice injected with AsSn cells. These details clarify the role of Snail in the regulation of RhoA, which is correlated with tumor metastasis by affecting cell movement.

A previous study indicated that the use of RNA interference may be an effective tool for blocking Snail function (22). We have also reported a strategy of combining antisense apoptosis-associated cDNA with an oncolytic adenovirus (23) and it appears that arming an oncolytic adenovirus with siRNA is also reliable in cancer gene therapy (24). Future studies should apply these methods progressively to Snail-targeted cancer gene therapy.

In conclusion, the present data support a novel role for Snail in the progression of breast tumors and provide evidence that this effect is mainly mediated through the regulation of RhoA activity which is involved in cell movement and growth *in vivo*. Based on these findings, Snail may be considered, in the future, as a putative molecular target for antineoplastic therapy.

## Figures and Tables

**Figure 1.** Expression of Snail and RhoA in breast tumors and normal breast tissues. (A) Immunohistochemical study using anti-Snail and anti-RhoA antibodies (breast cancer magnification, ×400; normal breast tissue magnification, ×200; scale bar, 40 *μ*m). (B) Western blot analysis demonstrating the higher expression of Snail and RhoA in breast tumors (T1, T2, T3) compared with corresponding normal breast tissue (N1, N2, N3).

**Figure 2.** AsSn transfection alters the EMT phenotype *in vitro*. (A) MDA-MB-231 and MDA-MB-435S cells were stably transfected with the AsSn. Mock-transfected cells served as controls. AsSn cells exhibited a clear decrease of Snail and RhoA expression; fibronectin and MMP-2 expression decreased by ∼30% compared with mock-transfected cells; and E-cadherin expression was induced. (B) Slug mRNA expression detection in AsSn- and mock-transfected cells by real-time PCR. No significant changes in the level of endogenous Slug mRNA were detected in AsSn- and mock-transfected clones. (C) Morphology of AsSn- and mock-transfected cells analyzed by phase-contrast microscopy. Mock-transfected cells remained spindle shaped, while AsSn cells exhibited a cobblestone-like morphology (original magnification, ×400). AsSn, antisense-Snail cDNA construct; EMT, epithelial-mesenchymal transition.

**Figure 3.** AsSn transfection inhibits cell motility *in vitro*. (A) Wound-healing ability of AsSn cells vs. mock-transfected cells. Mock-transfected cells frequently migrated into the wound area and filled in the wound after 24 h, whereas the AsSn monolayer migrated slowly into the wound. (B) Cell migration was estimated by means of Transwell migration assays. The numbers of migrated cells were estimated 10 h after seeding, then migrated cells were fixed, stained and photographed. The experiment was repeated three times. The invasion ability of the AsSn cells was significantly lower than that of the mock-transfected cells (P<0.05 for both). (C) Growth curves showing that there was no difference between the mock-transfected and AsSn cells in cell growth until 72 h after seeding. AsSn, antisense-Snail cDNA construct.

**Figure 4.** AsSn alters RhoA expression and activity, correlating with cell invasion. (A) Transient transfection of AsSn results show two to three-fold repression of RhoA promoter activity by Snail downregulation. (B) RhoGTPase levels in the lysates of mock-transfected and AsSn cells were analyzed by western blotting with β-actin serving as a quantitative control. The activities of the enzymes were determined by a pull-down assay using GST-C21 to detect Act-RhoA or with GST-PAK-CD for active Rac1 and Cdc42. Overexpression of AsSn led to a significant decrease of RhoA activity. (C) Mock-transfected and AsSn cells were transfected with expression vectors coding for the Wt, DN or Act forms of RhoA-GFP fusion proteins or GFP alone (GFP). Two days after transfection, cells were subjected to a Matrigel invasion assay. DN-RhoA significantly augmented the inhibitory effect of AsSn in cell invasion (*P<0.05). (D) Cells were lysed to assess the expression of fusion proteins by immunoblotting with anti-GFP or anti-RhoA antibody. (E) Mock-transfected and AsSn cells were transfected with expression vectors coding for Wt- or DN-RhoA-GFP fusion proteins. Two days after transfection, cells were lysed and subjected to immunoblotting with anti-MMP-2 antibody. MMP-2 expression and activity was decreased in cells transfected with DN-RhoA and increased in cells transfected with Act-RhoA. AsSn, antisense-Snail cDNA construct; Wt, wild-type; DN, dominant-negative; Act, active.

**Figure 5.** Effects of AsSn on tumorigenesis and angiogenesis in BALB/c SCID mice *in vivo*. (A) AsSn inhibited tumor growth. (B) Effects of AsSn on animal survival and associated gene expression in BALB/c SCID mice *in vivo*. The mice were euthanized and sacrificed when they appeared moribund or at the end of the observation period (90 days). (C) AsSn inhibited lymph node metastasis. Red arrows show lymph metastasis. (D) Western blotting analysis demonstrated that Snail and RhoA levels decreased significantly in tumors from mice injected with AsSn cells compared with mock-transfected cells. AsSn, antisense-Snail cDNA construct.

**Table I.** Snail and RhoA expression in normal breast and breast tumor.

Factor	No. of cases	-	+	Snail staining			RhoA staining				P-value
				++	+++	P-value	-	+	++	+++	
Normal breast	20	8	11	1	0	0.000	10	9	1	0	0.000
Breast tumor	60	5	8	15	32		3	7	30	20	

Snail and RhoA staining was scored as negative (-), weak (+), moderate (++) or strong (+++).

**Table II.** Clinicopathological association of Snail and RhoA expression in patients with breast cancer.

	No. of cases	Snail staining					RhoA staining				
		-	+	++	+++	P-value	-	+	++	+++	P-value
Differentiation						0.848					0.020
Well	12	2	4	4	2		1	5	4	0	
Moderately	18	2	3	5	8		2	2	3	3	
Poorly	30	3	9	10	8		2	3	18	7	
TNM						0.079					0.169
I+II	24	3	8	7	6		2	6	8	8	
III+IV	36	4	5	10	17		2	4	13	17	
Metastasis											
With	40	5	6	11	18	0.164	2	5	15	18	0.235
Without	20	2	7	6	5		2	5	6	7	

Snail and RhoA staining was scored as negative (–), weak (+), moderate (++) and strong (+++).

## Abbreviations:

AsSn: antisense-Snail cDNA construct;
DMEM: Dulbecco’s minimum essential medium;
EMT: epithelial-mesenchymal transition;
HMEC: human mammary epithelial cells
